The article "DNA barcoding identification of Pseudococcidae (Hemiptera: Coccoidea) using the mitochondrial COI gene" was retracted in 2019. Reasons: errors in the data; errors in the methods; unreliable data.

# DNA barcoding identification of Pseudococcidae (Hemiptera: Coccoidea) using the mitochondrial COI gene

**DOI:** 10.1080/23802359.2018.1457988

**Published:** 2018-04-04

**Authors:** Sizhu Zheng, Yang Li, Xiaojun Yang, Jingyun Chen, Jing Hua, Yuan Gao

**Affiliations:** a Suzhou entry exit inspection and Quarantine Bureau, Suzhou, Jiangsu Province, P.R. China;; b Jiangsu Entry- Exit Inspection and Quarantine Bureau, Lab for plant quarantine, Nanjing, Jiangsu Province, P.R. China

**Keywords:** Phenacoccus, Pseudococcus, *Planococcus*, identification, genetic distance

## Abstract

DNA barcoding is a recently developed technique for species-level identification that involves the use of short, standard DNA sequences as species labels. It is an effective complement to traditional taxonomic classification based on morphology. At present, research and applications involving the DNA barcoding of the Pseudococcidae are focused primarily on the cytochrome coxidase subunit I (*COI*) gene, but there is not yet a consensus on the preferred gene region for barcoding. The purpose of this study was to explore the effectiveness of identification of Pseudococcidae beetles using DNA barcoding technology. The *COI* gene sequences of 97 samples from 21 species of Asemini were analysed, followed by evaluation of the ability to identify species using a tree-building method and distance evaluation. The *COI* sequences (500 bp) exhibited distinct distributions of intra-specific and inter-specific variation and a significant barcoding gap. The success rate of identification was 97.84%. These results demonstrate the feasibility of using this segment of *COI* to identify most species of Pseudococcidae.

Mealybug is a kind of wide distribution, multi-host phytophagous insect, only a small part are resource insects, mostly are severe pests in the agriculture and forestry industry (Ben-Dov 2012). Morphological identification of Pseudococcidae species requires a long time and a high level of taxonomic expertise. Usually, only adult females can be identified. Besides, the traditional morphological identification has a limitation, which must require complete adults for study because of the difficult identification of the relative species, early morphological structures (eggs, larvae and pupae) and fragmentary bodies (Kondo 2008; Utsugi 2011).

With the development of molecular biology research, more and more technologies are applied for the identification of Pseudococcidae species (Zheng et al. 2015a, 2015b). The characteristic which is fast, accurate and automated for species identification by DNA barcoding allows the classification and identification of Pseudococcidae. More and more research staffs join the study of DNA barcoding, so that the field becomes a hotspot of biological study (Hebert 2003; Wei et al. 2015).

The mtDNA *COI* gene of insects becomes one of the most common molecular markers in insect taxonomy as a result of its maternal inheritance, high stability and conservation including enough variation at present. For example: ‘Moreover, the mtDNA *COI* sequences of Pseudococcidae reveal an higher variability than other genes in *Planococcus ficus*, *P. minor* and *P. citri*a and notably than 18S and 28S gene sequences (He et al. 2007). Park et al. (2011) revealed the characteristic of the nucleotide composition in scale insects DNA barcode sequences by redesigning the forward primer of *COI* gene sequences for the effectiveness study of the species identification in Diaspididae and Pseudococcidae. Saccaggi et al. (2008) distinguished *Planococcus ficus*, *P. citri* and *Pseudococcus longispinus* by the characteristic analysis of the mtDNA *COI* gene sequences.’ However, these data were still inconclusive, could not meet the requirements of accurate identification in Pseudococcidae species. The present study focused on 21 species of Pseudococcidae beetles. Our objective was to develop an accurate, rapid and practical method for identification of Pseudococcidae species using DNA barcodes. We developed a DNA barcode library for these 21 Pseudococcidae species by sequencing specimens from geographically distinct locations around the world. The utility of the DNA barcoding approach for identification of these Pseudococcidae species was assessed by computing intra- and inter-specific divergences, evaluating the barcoding gap and constructing phylogenetic trees.

## Method

### Specimens and DNA extraction

In this study, the samples were all preserved in 100% ethanol, including 93 individual samples which represented four families and 21 Pseudococcidae species, each sample had been sequenced three times to check the accuracy. All the sequences had been uploaded on Genbank and get the gene sequence numbers (Table 1). Meanwhile, in order to increase the quantities and species of gene samples and increase the scope of identification, we downloaded partial sequences from NCBI according to the location of primer sequences to improve the credibility of experimental results.

**Table 1.** Squences details and GenBank accession numbers.

Species names	GenBank accession numbers	Location
*Dysmicoccus brevipes*	KP981104	Philippines
*Dysmicoccus lepelleyi*	KP981101∼ KP981103	Malaysia
*Pseudococcus comstocki*	KP981091	China (Hangzhou)
*Pseudococcus jackbeardsleyi*	KP981087	Thailand
*Planococcus kraunhiae*	KP981070; KP981072	Japan
*Phenacoccus solani*	KP981073; KP981074; KP981088; KP981089	China (Suzhou)
*Phenacoccus solenopsis*	KP981092; KP981098	China (Suzhou)
*Phenacoccus solenopsis*	KP981093; KP981094 KP981096; KP981097	China (Gaungdong)
*Phenacoccus solenopsis*	KP981099	China (Hangzhou)
*Dysmicoccus brevipes*	HM47414;JN128961∼ JN128963	NCBI
*Dysmicoccus neobrevipes*	JN128958; JN128959	NCBI
*Phenacoccus aceris*	GU936935;HM474254; HM474255; HM474258 ∼ HM474262;	NCBI
*Phenacoccus avenae*	HM474263	NCBI
*Phenacoccus parvus*	JQ085560;KJ676517	NCBI
*Phenacoccus solani*	GU936937;HM474269	NCBI
*Phenacoccus solenopsis*	AB858432	NCBI
*Planococcus citri*	HM474278; HM474279; HM474283; HM474288	NCBI
*Planococcus ficus*	HM474290∼ HM474293	NCBI
*Planococcus kraunhiae*	GU936934;HM474302; HM474303	NCBI
*Planococcus lilacinus*	HM474307;HM474309; HM474310;KU254159	NCBI
*Planococcus minor*	HM474319;HM474320;KU254175;KU254176;KU254180	NCBI
*Planococcus vovae*	JQ085557	NCBI
*Pseudococcus baliteus*	KU056829∼ KU056835	NCBI
*Pseudococcus comstocki*	HM474366;HM474368; HM474387; HM474388	NCBI
*Pseudococcus calceolariae*	HQ179895∼ HQ179898	NCBI
*Pseudococcus cryptus*	HM474369∼ HM474373	NCBI
*Pseudococcus jackbeardsleyi*	HQ179901∼ HQ179903	NCBI
*Pseudococcus longispinus*	HM474377; HM474381; HM474386; HM474389; HM474391	NCBI
*Pseudococcus viburni*	HQ179909; Q179910; JQ085550; JQ085551;KJ530623	NCBI

After photographing, DNA template were extracted from the samples identified by morphology, 2 ∼ 4 whole mealybugs (<30 mg) for genome extraction. We used the GenMagBio animal magnetic tissue/cell genomic DNA extraction kit (GenMag Biotechnology Company, Beijing) according to the manufacturer protocol to extract DNA from samples (Zheng et al. 2012; Wei et al. 2015).

The final DNA extract was preserved at 4 °C.

#### DNA amplification and sequencing

A target 650-bp fragment of *COI* was amplified by polymerase chain reaction (PCR) using an Eppendorf Mastercycler pro and following primers: PcoF1-5′-CCTTCAACTAATCATAAAAA TATYAG-3′ and LepR1-5′-TAAACTTCTGGATGTCCAAAAAATCA-3′ (Park et al. 2011). The amplification protocol was set as follows: 95 °C for 4 min; followed by 35 cycles at 94 °C for 1min, 48 °C for 1min, and 72 °C for 45 s; and a final extension at 72 °C for 4 min. PCR products were separated by electrophoresis on a 1.5% agarose gel containing ethidium bromide and then visualized and photographed under ultraviolet transillumination prior to clean up and sequencing. Successful PCR products were sent for sequencing at the Genewiz Biotechnology Company (Jiangsu, Suzhou, China) using the aforementioned primers.

#### Data processing

Altogether we obtained sequences from 93 individuals. Original chromatograms of sequences were manually checked to avoid reading errors and the low-quality ones were excluded from further analysis. After assembling, products were cut to a final 500 base pair fragment of *COI* gene. Sequences from each locality were aligned and all the identified haplotypes were submitted to GeneBank. These analyses were performed in DNAStar or BioEdit (Pettengill et al. 2010). Spliced sequences were verified against sibling species using the BLAST program from NCBI. A neighbour-joining (NJ) tree was created, and sequence lengths, GC contents, polymorphic sites and genetic distances were calculated using Mega 5.05 (Tamura et al. 2011). The pairwise summary module in TaxonDNA (Meier et al. 2006) was used for determining the barcoding gap, the Distance Analysis module was used to compute interspecies genetic distances, and the Best Match and Best Close Match modules were used to compute the efficiency of species identification.

## Results

### *Sequences characteristic of pseudococcidae* COIs

We found no deletions or insertions in any of the sequences from GenBank or in any of the sequenced samples. All sequences were implemented into Mega 5.0 as equal-length segments of 500 bp, including 206 variable sites, 294 conserved sites, 192 parsimony-informative sites, and 14 singleton sites. The average A, G, C and T were 35.0%, 5.1%, 11.0% and 48.9%, respectively. The A + T content was 83.9%, considerably higher than the G + C content, indicating an A + T preference. In addition, the A content was equal to the T content, reflecting a similar pattern of nucleotides composition to that of the mitochondrial DNA of other insects. The overall transition/transversion (ts/tv) ratio was 0.5, and a high ts/tv ratio was found at the first codon position (1.34). The first codon position was most conserved and exhibited a high ts/tv ratio, as observed in other studies on beetles (Stauffer 1997).

### Genetic divergence within and between species

Table 2 shows partial sequence divergences among and within species using Kimura’s 2-parameter (K2P) genetic distance method. The results showed that average intra-specific K2P divergence for *COI* was 0.00825, ranging from 0.0 to 0.08. The intra-specific K2P divergence of *Pseudococcus comstocki* was highest. Inter-specific K2P divergences ranged from 0.02 to 0.214, with an average of 0.0978. The highest inter-specific K2P divergence was observed between *Phenacoccus aceris* and *P. parvus*, ranging from 0.195 to 0.214. The inter-genus ranged from 0.063 to 0.188 appeared between *Dysmicoccus* and *Planococcu*s. The difference between the maximum intra-specific and minimum inter-specific divergence is known as the barcoding gap (Figure 1). Two distinct distributions were observed for intra- and inter-specific variation of the *COI* gene with little overlap and distinct gaps. This indicates that the amplified sequences were suitable for distinguishing Pseudococcidae species.

**Figure 1.** Revised barcoding gap between interspecific and intraspecific divergences among samples for species identification based on the phylogenetic gene.

**Table 2.** The statistical results of Inter-specific distance, Intra-specific distance (%).

Gens	Intra-specific distance			Inter-specific distance		
	Minimum	Maximum	Average	Minimum	Maximum	Average
*Dysmicoccus*	0	2.0	0.7	8.9	13.6	8.3
*Phenacoccus*	0	5.6	0.8	6.5	21.4	13.5
*Planococcus*	0	1.0	0.2	2.0	11.7	8.0
*Pseudococcus*	0	8.0	1.6	3.7	15.0	10.5

### Phylogenetic analysis

A phylogenetic tree was built using the neighbour-joining (NJ) method based on Kimura’s 2-parameter model. Bootstrap values for individual clades were calculated by running 1000 bootstrap replicates of the data (Figure 2). Outgroup species were *Unaspis yanonensis* (KP981078, KP981079). We only considered queries to be correctly identified if they were found in a species-specific polytomy or at least one node into a clade exclusively consisting of sequences from one species. A query was considered ambiguous if it was determined to be a sister group to a cluster of conspecific sequences of a different species. Results showed that different geographical populations of 21 species of Pseudococcidae clustered together as one clade in the NJ trees without overlapping .Sequences belong to the same genus clustered into one group which are clearly split and genetically relatively distant from each other. The sequences of the 21 species supported the traditional taxonomy at the genus and species levels.

**Figure 2.** The Neighbour-joining tree for 21 species of Pseudococcidae based on *COI* sequences. Note: The numbers at the nodes indicate the bootstrap values, and only values above 50% are given. Scale bar indicates the genetic distance.

### Identification effect of COI gene on pseudococcidae species

We used the Best Match module in TaxonDNA to find its closest barcode match for each sequence. If the sequences all belonged to the the same species, the identification was considered a success, whereas mismatched names were counted as failures. Several equally good best matches from different species were considered ambiguous. According to the 5.4% threshold based on the intra-specific genetic distance, we conducted those sequences as no match that had no matching sequences found (Meier et al. 2006). The identification successful rate of *COI* gene in the Pseudococcidae species was 97.84% (Table 3). The result demonstrate that this *COI* gene fragment of 500 bp can be used to accurately identify most species of Pseudococcidae.

**Table 3.** Identification success rate (%) based on ‘Best match’ and ‘Best close match’.

Best match			Best close match			
Successful identification	Ambiguous identification	Misidentification	Successful identification	Ambiguous identification	Misidentification	No match
97.84%	0%	2.15%	97.84%	0%	0%	2.15%

## Discussion and conclusion

DNA ‘barcode’ usher a new era for the identification of Pseudococcidae. Reliable species identification is essential measure of DNA barcoding which should meet important criteria such as a short DNA region allowing amplification of degraded DNA. Second, it should be sufficiently variable to distinct different species, conserved enough to be less variable within than between species. Third, the target DNA region should contain enough phylogenetic information to easily assign species to its taxonomic group (genus, family, etc.) (Taberlet et al. 2007). In this study, the length of *COI* gene fragment we used was 500 bp, which reduced the demand on the quality of samples, had high amplification efficiency. The average intra- and inter-specific K2P genetic distance of 21 species of *Pseudococcidae* was 0.825% and 9.78%, the average inter-specific genetic distance was ten times (10×) more than the average intra-specific genetic distance, which indicated that the *COI* gene fragment could be used as identification of Pseudococcidae species (Hebert et al. 2003).

We used K2P distance method and tree construction to evaluate the identification of *COI* gene and corresponding species. The result indicated that this *COI* gene could identify the Pseudococcidae species and the success rate reached 97.84%. The success rate of *Planococcus vovae* and *Phenacoccus avenae* cannot be calculated, because their different geographical populations could not be found. The sequences belonged to different geographical populations of other *Pseudococcidae* species clustered into one group without overlapping and with well-support bootstraps, which supported the traditional morphological classification.

Not only DNA barcoding can be used as identification of species, but also can help us having acquaintance of phylogenetics. Of the samples included 21 species representing 4 genus, the average intra-specific genetic distance of *Pseudococcus comstocki*, *P. longispinus*, *Phenacoccus aceris*, *Planococcus ficus* was 4.6%, 3.4%, 4.2%, 2.2% (>2%), which indicated that the four species had begun to have a disproportionation. The exception was *Phenacoccus aceris* and *P. parvus*, whose K2P distance was 0.195 to 0.214 and inter-specific genetic distance appeared to be the largest, far more than the genetic distance of genus between *Phenacoccus* and three other genus, of which illustrated that geographical isolation made the two *Phenacoccus* species more divergent.

For the study of DNA barcoding of insect taxa, mitochondrial cytochrome c oxidase I (*COI*) gene has been widely used. In the study of *Pseudococcidae* species, the *COI* gene fragment we obtained whose length is 500 bp, is easily amplified. It has a high success rate of identification and a comparatively high practical value.
